The article "Construction of Game Model between Carbon Emission Minimization and Energy and Resource Economy Maximization Based on Deep Neural Network" was published in 2022. Journal: Comput Intell Neurosci.

# Construction of Game Model between Carbon Emission Minimization and Energy and Resource Economy Maximization Based on Deep Neural Network

**DOI:** 10.1155/2022/4578536

**Published:** 2022-05-02

**Authors:** Lan Ma, Dalei Wang

**Affiliations:** ^1^School of Math and Statistic, Suzhou University, Suzhou, Anhui 23400, China; ^2^School of Mechanical and Electronic Engineering, Suzhou University, Suzhou, Anhui 23400, China

## Abstract

Under this background, this paper tries to find countermeasures and ways for carbon reduction by observing and analyzing the influencing factors of carbon emissions, designing ways to minimize carbon emissions and maximize resources and energy. In view of the above problems, the carbon emission prediction research is closely combined with the research of deep neural network, the carbon emission prediction models based on deep neural network are established, respectively, and the game theory is introduced to maximize the resource economy. Based on the analysis of the cost of energy resources, this paper puts forward a model based on game theory and makes an overall planning of the bidding online auxiliary decision-making system in combination with the actual market demand. Build a big data analysis platform based on the Internet of things, collect the data related to carbon emission for normalization, analyze the influencing factors related to carbon emission by using the principal component analysis method, select the data with higher connection value, and take the time series data as the input of the deep neural network for simulation verification. The simulation results show that the game model of carbon emission minimization and energy resource economic maximization based on deep neural network can effectively improve the economic maximization of energy resources and reduce carbon emissions.

## 1. Introduction

Statistics show that energy consumption in various countries is increasing year by year, and people's quality of life has also been significantly improved [1]. This is mainly due to the rapid development of economic globalization. As the largest developing country in the world, China's climate change trend is consistent with the global climate change trend [2]. The enhancement of the global greenhouse effect has attracted extensive attention of various organizations and countries. A large amount of carbon dioxide emission is one of the reasons for the strengthening of the global greenhouse effect. Reducing carbon dioxide emission can effectively avoid the greenhouse effect [3]. The academic circles at home and abroad focus on the issue of carbon emission, which has won the strong support of governments all over the world. Facing this long-term and urgent carbon reduction goal, China has actively made response measures and put forward methods and ways to effectively reduce carbon dioxide emissions per unit of GDP [4–6].

A large number of scholars have invested in carbon emission research, which is a new topic, involving a variety of methods [7–9]. Through the research on foreign carbon emission research, it is found that the research on carbon emission mainly involves quantitative model analysis, and there are many studies on carbon emission using STIRPAT model [10]. Literature [11] describes that the traditional economic model EE is improved to obtain STIRPAT model. When STIRPAT model is used in carbon emission research, it is developed into IPAT and IM IPAT models. The advantages and disadvantages of this model are different. When studying carbon emissions in different regions, it is necessary to carefully analyze the applicability of H models in data fitting. Literature [12] has conducted in-depth research on the low-carbon industrial chain, combined qualitative research with quantitative research, and constructed a set of evaluation index system to measure whether the industrial chain has achieved low-carbon development, which provides a certain guiding significance for the development of low-carbon economy in China. In [13], through the research on low-carbon economy at home and abroad in recent years, it is found that the research direction of low-carbon economy is more detailed and gradually specific to the enterprise level, and the empirical research method is more and more favored by researchers. Literature [14] points out the opportunities and challenges faced by China in developing low-carbon economy, analyzes the problems that may be encountered in the process of developing low-carbon economy in the future, and puts forward countermeasures. Literature [15] studies the carbon emissions of low-income countries, middle-income countries, and high-income countries and uses STIRPAT model to analyze the impact of different factors on carbon emissions of countries with different income levels. The research shows that the per capita GDP level and energy intensity have a great impact on low-income countries and middle-income countries, respectively, while the factors show a great positive correlation in high-income countries. Literature [16] analyzes the impact of the main emission of greenhouse gases and energy consumption on China's environment and makes a quantitative study of China's data from 1978 to 2016 by using STIRPAT model. The analysis shows that population factors have the greatest impact on the environment, including urbanization level and industrial level. Literature [17] analyzes the carbon emissions of developed countries and establishes STIRPAT model. It is found that the factors affecting the carbon emissions of developed countries are not only population, per capita wealth, and energy intensity, but also energy structure, residents' energy consumption, and urbanization rate. It is pointed out that the STIRPAT model needs to be adjusted appropriately when studying the carbon emissions of different countries,and W gives better results. Literature [18] analyzes the five factors affecting China's carbon emissions. It is found that the influence degree of the five factors on carbon emissions is per capita GDP, technical level, population, urbanization rate, and industrial structure, and the technical level is the most effective solution in energy conservation and emission reduction. Literature [19] studies the influencing factors of China's energy demand through integration analysis of energy demand factors. The research results show that the major factors affecting energy demand are energy intensity, energy structure, urbanization level, population, industrial structure, and energy price. Literature [20] studies China's direct domestic carbon emissions and decomposes the influential factors into five factors: energy structure factor, carbon emission coefficient factor, consumption energy intensity factor, per capita consumption level, and family size and quantitatively analyzes these factors [21]. According to China's current carbon emission policy, considering the impact of introducing consumers' low-carbon consumption preference under the two policies of independent emission reduction and mandatory emission reduction, this paper studies the impact of different strategies adopted by supply chain enterprises in carbon emission reduction on their production and operation and discusses the optimal strategy of carbon emission in supply chain through comparative analysis. The main contributions are summarized as follows.

In order to minimize carbon emissions and maximize resources, this paper establishes a resource monitoring platform based on IOT and designs the cloud network platform structure based on the Internet of things. In addition, this paper establishes a carbon emission prediction model based on deep neural network. In order to improve the training speed of the network, the principal component analysis method is used to reduce the dimension of the original data. Taking the processed data as the input of the neural network model, the optimal carbon emission prediction can be obtained. According to the carbon emission prediction model and considering the maximization of resource economy, a game model of resource economy is established. Finally, the effectiveness and reliability of the model are verified by simulation.

## 2. Architecture Design of Data Platform Based on IoT

### 2.1. Overall Structure Design of System Architecture

With the progress of the times, a large number of facilities and equipment with real-time communication function are applied to the observation network, resulting in the storage, transmission, and integration of massive multivariate and heterogeneous data and the in-depth mining of data information, which has expedited the development of two technologies, data center and Internet of things, and pushed human society into the digital era. Internet of things and data center technology have shown many advantages that traditional technologies do not have in recent years. For example, the Internet of things can realize real-time transmission of accurate and multidimensional data information in the full coverage field; the data center station can provide stable and standardized data services in a complex and multisource data environment, which provides a strong technical guarantee for the construction of an integrated platform for the comprehensive observation of natural resource elements.

As shown in Figure 1, the data center is the core of the construction of comprehensive observation data resource system, mainly including observation data resource directory, data model construction, data standardization and integration, and database and data linkage update. The comprehensive observation data resource catalogue is the basis for the interconnection, sharing, and exchange of natural resource data. The scope of the resource catalogue covers the data of primary, secondary, and tertiary observation stations, including basic support data, element observation data, element thematic product data, and system maintenance data by combining the data resources of comprehensive observation of natural resources, analyzing the levels, categories, and relations between the data, making a unified planning for the data resources in the field of comprehensive observation of natural resource elements, and formulating a unified data resource coding and classification system. Among them, the element observation database mainly includes Internet of things data, basic database, and decision analysis database, involving massive structured data and unstructured data. Therefore, the hybrid storage mode of relational database and distributed system is adopted to realize the storage and management of big data of natural resources. The distributed architecture part is used to store offline massive structured data, semistructured data, and unstructured data, and the traditional relational database part is used to store structured data with small amount of data. Because the query and processing speed is high, and the required storage space is only half of the traditional relational database, the time series database is used for the massive stream data, time series data, and monitoring data of the Internet of things.

In addition, as a new architecture of data interface, the function of data middle station technology is to standardize the increasingly large and multichannel observation data information such as resources and population, separate the data from the application interface, and then calculate and process. The data center is related to every link in the natural resource element observation data system, such as data generation, collection, transmission, storage, sharing, use, and update. The data system is divided into four levels: the post source data layer is mainly composed of comprehensive observation data of natural elements, original accumulated data, and shared data of other stations and networks; the tag data layer is composed of manager tag, researcher tag, and user tag. The data analysis application layer mainly corresponds to the top-level service object of the integrated platform and is oriented to resource asset management applications and scientific research data sharing applications; data service engine mainly includes data query service, real-time data service, data analysis service, and batch data service; the unified data layer mainly includes information data, scientific research information data, dataset information data, and personnel information data.

### 2.2. Structure Design of Cloud Platform Based on IoT

Internet of things center is an important way for data transmission to enter the data center of natural resource elements. The Internet of things center provides functions such as connection management, equipment management, perceptual data management, system management, and security management. Through the unified access and management of sensors, and the unified processing of their own information such as sensor location and status, as well as the information obtained by sensors, it provides perceptual decision-making data support for comprehensive business applications.

As shown in Figure 2, the data processing platform based on cloud computing is also a mining link in the data processing of the Internet of things. In the model, the parallel operation and distributed operation of mining algorithm and recommendation algorithm are fully considered. The model divides the data processing platform into three basic levels. The idea of hierarchical design makes the whole Internet of things data processing more effective and the processing efficiency has been greatly improved. From bottom to top, there are the cloud computing support platform layer, data mining capability layer, and data mining cloud service layer. Furthermore, the model cloud technology refers to building a set of model service platform based on “cloud,” fully considering the interaction between resources, and forming a model computing platform integrating all services such as spatial structure analysis, bearing capacity suitability evaluation, action mechanism analysis, and coupling balance research of various natural resources. It mainly includes cloud model computing platform and local business access system. Cloud platform also includes front-end service, scheduling service bus, model operation virtualization container, and shared data service.

## 3. Research on Carbon Emission Minimization and Energy and Resource Economy Maximization Based on Deep Neural Network

In order to minimize carbon emissions and maximize resource economy, the overall framework of the algorithm is designed in Figure 3. As shown in Figure 3, the algorithm framework mainly includes data sources, data dimension reduction, carbon emission prediction, resources maximization game, and data visualization.

### 3.1. Research on Data Dimension Reduction Based on PCA Method

Principal component analysis (PCA) is a commonly used dimensionality reduction method in multivariate statistics. At present, PCA has been successfully applied in many research fields, such as power system coherent cluster identification, state estimation, load forecasting, and transformer fault diagnosis. Its basic idea is to use fewer unrelated new variables (indicators) to replace the original more related variables (indicators), and the new variables are the linear combination of the original variables. The selected new variable is called the main component, and the selection principle is to retain the information contained in the original variable as much as possible. From the perspective of statistics, the information contained in a variable can be characterized by its variance. The greater the variance, the greater the amount of information contained.

The essence of principal component analysis is the translation and rotation of coordinates. Suppose that there is a two-dimensional data table. The schematic figure PCA algorithm is shown in Figure 4. The problem of the original two-dimensional data space can be simplified to one-dimensional data space for analysis. The idea is also valid when it is extended to high-dimensional space.

Let the index data composed of *n* planning schemes and *p* evaluation indexes be *X*=(*x*_*ij*_)_*n*×*p*_ where *x*_*ij*_ is the value of the *j*-th index of the *i*-th scheme. The index data is standardized by the following equation:

(1) $$\begin{array}{c} z_{ij}=\frac{x_{ij}-{\bar{x}}_{j}}{{\bar{s}}_{j}}, \end{array}$$

where ${\bar{x}}_{j}$ and ${\bar{s}}_{j}$ are the mean and mean square deviation of the *j*-th index value, respectively. Then, establishing the correlation coefficient matrix of standardized data *R*=(*r*_*ij*_)_*p*×*p*_， the element *r*_*ij*_ in the matrix reflects the correlation between the index *z*_*i*_ and *z*_*j*_.

(2) $$\begin{array}{c} r_{ij}=\frac{\text{Cov}\left(z_{i},z_{j}\right)}{\sqrt{D\left(z_{i}\right)}\sqrt{D\left(z_{j}\right)}}, \end{array}$$

where Cov(*z*_*i*_, *z*_*j*_) is the covariance of indexes *z*_*i*_ and *z*_*j*_. In addition, the correlation coefficient matrix is equal to the covariance matrix, which can be obtained by using the following formula:

(3) $$\begin{array}{c} R=\frac{1}{n-1}Z^{T}Z, \end{array}$$

*λ*_*i*_ is the variance of the principal component *y*_*i*_. The contribution rate of the variance of principal component *y*_*i*_ to the total variance is

(4) $$\begin{array}{c} w_{i}=\frac{\lambda_{i}}{\sum_{j=1}^{n}\lambda_{j}}, \end{array}$$

The contribution rate *w*_*i*_ reflects the percentage of the *i*-th principal component carrying the original variable information. Therefore, the variance contribution rate of the first principal component is the largest and decreases step by step.

### 3.2. Carbon Emission Prediction Model Based on Deep Neural Network

In recent years, many scholars have done different research on carbon emission prediction for different objects [22, 23]. At present, the existing research results mainly focus on carbon emission prediction for power industry, province, city, or single region. Based on China's total carbon emission and influencing factors in recent 33 years, this paper trains different network models for prediction and analysis, There is a slight innovation in the research object. In addition, this paper carries out grey correlation analysis on a variety of different influencing factors of carbon emission, determines the main influencing factors, and uses different neural network models for prediction and analysis, which not only compares the prediction performance between different neural network models, but also analyzes the prediction results of carbon emission and gives the corresponding carbon reduction countermeasures and suggestions.

The process of nonlinear function fitting algorithm based on deep neural network can be divided into three parts: deep neural network construction, deep neural network training, and deep neural network prediction, as shown in Figure 5.

As shown in Figure 5, the model construction of deep neural network is the most important in the whole process. The construction of deep neural network includes the selection of neurons, the number of hidden layers, and the number of neurons between layers.

Therefore, the network structure design of convolution layer is the core of the whole deep neural network. In order to achieve high-precision prediction, this paper designs the convolution network design as shown in Figure 6.

The first layer of the convolution neural network is the convolution layer, which uses some adjustable parameter patterns as filters to convolute the input data. Convolutional neural network was initially applied to the research of some computer vision directions. For example, in handwriting recognition, *w* can automatically learn the features of edges, corners, or curves of the input image. Similarly, in the specific search and prediction of biological gene sequence, we also design a convolutional neural network to automatically learn fragment features. In fact, this method of using convolution neural network technology to realize prediction model can be easily extended to many useful directions. In addition, a 3 *∗* 3 pooling layer is used to optimize the data. Finally, two full connection layers are designed to recover data, and sigmoid function is selected to classify the data.

### 3.3. Research on Resource Maximization Based on Game Theory

Game theory is a theory that uses rigorous mathematical models to solve the conflict of interests in the real world. Because conflict, cooperation, and competition are common phenomena in the real world, game theory can be applied in many fields, such as military field, economic field, political and diplomatic resolution, such as tactical attack and defense, international dispute pricing, fixed production, merger, acquisition, bidding, auction, and even animals evolution and other issues.

Mandatory emission reduction (command and control) refers to emission reduction under the compulsion of the government's administrative order. Under this mechanism, the government is the manager of the carbon rights market and is responsible for allocating the initial quota of enterprises. Enterprises must complete the emission reduction tasks assigned by the government. They can achieve the emission reduction tasks through their own emission reduction or carbon trading market. If enterprises fail to meet the emission reduction targets imposed by the government, they will be severely punished by the government. In this paper, the carbon emission right initially allocated by the government to enterprises is taken as the amount of mandatory emission reduction by the government to enterprises. In this paper, IO is taken as the constraint condition of enterprise carbon emission; that is, when the enterprise's carbon emission is smaller than the government's initial quota, then the enterprise will certainly sell its own excess carbon emission in the carbon market. On the contrary, enterprises will avoid the punishment of the government through their own emission reduction and the purchase of carbon rights in the carbon market.

Therefore, the total carbon emission of enterprises is mainly composed of the quota initially allocated by the government, the amount of carbon rights saved through technological upgrading *τ*_*A*_*Q*, and the trading amount obtained through market trading is *E*_*t*(*i*)_. At the same time, based on the assumption of rational people, enterprises will seek to maximize profits, and the carbon quota of enterprises will be fully utilized, that is,

(5) $$\begin{array}{c} E_{A}=O_{A}+\tau_{A}\chi_{A}Q-\tau_{A}Q+E_{t\left(A\right)},\\ \pi_{A}=\left[P_{A}-c_{A}-\chi_{A}p_{c}\left(1-\tau_{A}\right)\right]\left[M+\beta \tau_{A}\right]+\\ +O_{A}p_{c}-0.5t\tau_{A}^{2}-0.5e. \end{array}$$

where *E*_*A*_ is the total carbon emission of upstream enterprise *A* in the supply chain; *χ*_*A*_ refers to the carbon emission per unit product of enterprise *A*; *p*_*c*_ represents the market carbon trading price; *Q* can be expressed as the decreasing function of product price and the increasing function of carbon emission reduction rate; *O*_*A*_ refers to the initial quota of carbon emission rights freely obtained by enterprise *A*; *π*_*A*_ means revenue. The overall profit function of energy resources can be expressed as

(6) $$\begin{array}{c} \pi =\left[\left(P_{A}+P_{B}\right)-\left(c_{A}+c_{B}\right)-\chi_{A}p_{c}\left(1-\left(\tau_{A}+\tau_{B}\right)\right)\right]\left[M+\beta \left(\tau_{A}+\tau_{B}\right)\right]+\\ +\left(O_{A}+O_{B}\right)p_{c}-0.5t\tau_{A}^{2}-0.5e. \end{array}$$

where *τ*_*A*_ is the emission reduction rate; *e* refers to the additional expenses incurred in the communication between enterprises; *c*_*A*_ represents the production cost of a single product produced by the manufacturer; *c*_*B*_ represents the selling cost of a single product sold by the seller; *M* represents the selling cost of a single product sold by the seller.

This paper uses game theory to maximize resource benefits. The block diagram of the algorithm is shown in Figure 7.

## 4. Experiment and Result Analysis

According to the research needs, first, set the scenario value of the input independent variable from 2010 to 2015, then use the trained depth neural network to predict, and finally give the carbon reduction countermeasures and ways according to the analysis of the prediction results. Using homogeneous neural network model to predict carbon emission intensity, one of the important assumptions is that the historical value of time series can be used to predict the future value. In addition, data is the basis of model prediction. The following will focus on the data sources.

Data on China's population, urbanization rate, per capita GDP, industrialization level, proportion of tertiary industry, energy structure, energy utilization rate, per capita GDP energy consumption, natural gas consumption, and nuclear power consumption from 1983 to 2012 were collected for model training. The data of China's population, urbanization rate, per capita GDP, industrialization level, proportion of tertiary industry, energy structure, energy utilization rate, energy consumption per unit GDP, natural gas consumption, and nuclear power consumption from 2012 to 2015 are used as the validation data set. Verify the effectiveness and reliability of the algorithm and model in MATLAB simulation environment.

The quality of indicators plays a decisive role in the prediction results of carbon emissions. The world carbon emission prediction indicators are complex and diverse. It is of great significance to select scientific and reasonable world carbon emission indicators. On the basis of Kaya formula, referring to relevant literature and according to the principle of availability and quantification of indicators, this paper selects economic, social, environmental, energy, and other factors as the primary indicators of world carbon emission prediction, which fully extracts the relevant information affecting carbon emission prediction and increases the accuracy of the fusion prediction model.

### 4.1. Data Dimension Reduction Analysis Based on PCA

Carbon emission is produced by a complex social and economic activity, and there are many influencing factors. Therefore, it is difficult to find out all the influencing factors when establishing the carbon emission intensity prediction model. However, the carbon emission intensity calculated according to historical data is the result of the interaction of all influencing factors, which implies the law of the impact of all influencing factors on carbon emission intensity. The dimensionality reduction analysis of the original data set is carried out through PCA, and the results are shown in Figure 8. As shown in the figure, among the seven influencing factors, GDP has the greatest impact on carbon emissions, with an influence coefficient of 1.12; that is, if GDP increases by 1.00%, the total carbon emissions will increase by 1.12% when other influencing factors remain unchanged. Secondly, the factor that has a great influence on carbon emissions is the proportion of the secondary industry, with an influence coefficient of 0.92; that is, for every 1.00% increase in the proportion of the secondary industry, carbon emissions will increase by 0.92%.

In order to reduce carbon emissions, Hebei Province should actively adjust the industrial structure, vigorously develop the tertiary industry and agriculture, reduce carbon emissions, and achieve sustainable development on the premise of maintaining rapid economic development. Population is also a major factor affecting carbon emissions.  Figure 8(b) shows dimension reduction analysis of the original data by the main principal component analysis method and analyzes the factors that have the greatest impact on resource emission. They are GPD, population size, and urbanization rate. There is also a positive correlation between them, but the influence coefficient is small, indicating that the total carbon emissions will increase with the increase of population. The influence coefficient of energy price on carbon emission is 0.12, indicating that if the energy price increases, the energy consumption will also increase, resulting in the increase of carbon emission, but the range is small, indicating that the demand for energy is not elastic. There are two main reasons: first, energy consumption is not replaceable. At present, people have no other alternative energy, and the price has little effect on its regulation. Second, although the price of energy such as coal and oil has been marketed, the price of electricity has not been fully marketed, and there is no significant negative correlation between electricity price and supply and demand. Therefore, the marketization of energy prices needs to be further promoted, especially the marketization of electricity prices, timely adjust electricity prices according to market demand, and give play to the role of price leverage; at the same time, we should actively promote the work of carbon emission tax, which can be piloted in key industries of energy consumption and gradually popularized after gaining experience. Urban structure is also the main factor affecting carbon emissions, and the influence coefficient is −0.47, indicating that there is a negative correlation between energy structure and carbon emissions; that is, with the development of diversified energy structure, carbon emissions decline.

### 4.2. Model Prediction Results Analysis Based on Deep Neural Network

According to the characteristics of carbon emission, wavelet neural network is designed. The network is divided into three layers: input layer, hidden layer, and output layer. Among them, the input layer input is five key factors affecting carbon emission; hidden layer nodes are composed of wavelet functions; the output layer outputs the carbon emissions in the predicted year. In wavelet neural network fitting, from the data of carbon emission and its influencing index factors from 1983 to 2015, the training span is 3, and the prediction output from 1990 to 2015 is predicted by iterative training, which is fitted with the actual value of carbon emission in the corresponding 30 years and analyzed for error.

The fitting effect and prediction performance of wavelet neural network are observed by visual method. The simulation results are shown in Figure 9. As shown in Figure 9, the fitting effect of the depth neural network is good, which can generally reflect the same trend of the predicted output and the expected output, and the average prediction error is significantly less than that of RBF neural network and wavelet neural network, which belongs to the normal prediction range and can reflect the strong prediction ability of the depth neural network.

In order to better illustrate the prediction ability of the model, the comparison between the predicted value and the actual value from 2010 to 2019 is shown in Table 1.

Table 1 shows the prediction results of the above three intelligent prediction models. In the long-term prediction of carbon emission prediction with a large time span, the growth rate of carbon emission varies greatly in different periods, and the key influencing factors on carbon emission in different periods are also different, and there are many influencing factors. Therefore, in the three prediction models, in order to better train the network and achieve the expected fitting accuracy and effect, the iterative training of training samples is adopted in the process to make the prediction effect approach the expected output continuously. Among them, RBF neural network can output better fitting effect, which roughly reflects the same trend of predicted output and expected output, and the average percentage of prediction error is close to 5%. However, wavelet neural network fails to achieve the expected effect, and the reason has been explained in the above summary.

### 4.3. Maximization Results Analysis of Resource Economy

Improve energy efficiency and reduce carbon dioxide emissions. The consumption of raw coal is not only the main source of energy carbon emissions, but also the main source of carbon dioxide. Moreover, the consumption proportion of raw coal is also large, and the carbon emission is significantly higher than that of natural gas and oil. Therefore, we should increase the proportion of natural gas, hydropower, and oil in the energy structure and change the phenomenon of coal dominated energy structure. In addition, from the perspective of long-term development of low-carbon cities, we should also accelerate the development of nuclear power and biomass power generation and further increase the proportion of clean energy such as nuclear power and biomass power generation. In the near future, on the premise that economic development and energy structure will not change rapidly, strictly controlling the growth of carbon emissions caused by energy consumption and improving energy efficiency is an effective measure.

Figure 10(a) depicts the comparison of the economic benefits and capabilities of various energy sources based on the game strategy. It can be seen that the stronger the proportion of clean energy, the higher the benefits.  Figure 10(b) depicts the comparison of the benefits generated under the three distribution strategies. Furthermore, it can be seen that, in most cases, the benefits generated based on the game strategy are greater than those generated by the conventional strategy.

## 5. Conclusion

This paper closely combines the research of carbon emission prediction with the research of deep neural network and establishes the carbon emission prediction model based on deep neural network. In the carbon emission prediction model, in order to achieve the expected fitting accuracy, this paper uses the principal component analysis method to reduce the dimension of the data with low correlation before training the samples and adopts the iterative training method. By comparing the fitting results, it is found that the depth neural network can better predict the carbon emission, compared with RBF neural network and wavelet neural network. In addition, based on carbon emission prediction, this paper establishes an economic maximization game model of energy resources to improve benefits. The simulation results show that the algorithm can effectively predict carbon emissions, keep the error within 5%, and have high prediction accuracy. Finally, the simulation analysis shows that the resource maximization model based on game theory can achieve the maximum benefit on the basis of maintaining the carbon emission limit and improve the influencing index factors of carbon emission prediction model. Due to the complexity of the carbon emission prediction system, its internal regularity needs to be revealed by a large number of empirical studies. Due to the single sample of the system, there will be some limitations in the model test. Therefore, in the future, it is necessary to conduct a large number of in-depth empirical studies on different samples to reveal the internal laws of the factors affecting the prediction of carbon emissions.

## Figures and Tables

**Figure 1:** System architecture design based on IoT.

**Figure 2:** Structure figure of cloud platform based on IoT.

**Figure 3:** Overall structure figure of algorithm.

**Figure 4:** The schematic figure PCA algorithm. (a) Original data before PCA processing. (b) Data after PCA processing.

**Figure 5:** Flowchart of carbon emission prediction model based on deep neural network.

**Figure 6:** Structure of convolution network design.

**Figure 7:** Algorithm framework diagram based on Game Theory.

**Figure 8:** Efficiency comparison of three semantic interaction strategies. (a) Data dimension reduction; (b) influencing factors analysis.

**Figure 9:** Comparison figure of model prediction results.

**Figure 10:** Income analysis based on Game Theory. (a)Income under different proportion of energy structure. (b) Income comparison.

**Table 1:** Comparison results between three models.

Network	MAE	Mean square deviation
Deep neural network	0.3802	0.0021
RBF neural network	3.5814	0.1653
Wavelet neural network	4.9875	0.2645

## Data Availability

The data used to support the findings of this study are available from the corresponding author upon request.
